RETRACTED

# Evolving Long Short-Term Memory Network-Based Text Classification

**DOI:** 10.1155/2022/4725639

**Published:** 2022-02-21

**Authors:** Arjun Singh, Shashi Kant Dargar, Amit Gupta, Ashish Kumar, Atul Kumar Srivastava, Mitali Srivastava, Pradeep Kumar Tiwari, Mohammad Aman Ullah

**Affiliations:** ^1^Computer and Communication Engineering, School of Computing and IT, Manipal University Jaipur, Jaipur, India; ^2^Department of Electronics and Communication Engineering, Kalasalingam Academy of Research and Education, Virudhunagar, Tamilnadu, India; ^3^Department of Electronics and Communication Engineering, Narasaraopeta Engineering College, Narasaraopeta, Andhra Pradesh, India; ^4^Department of Computer Science and Engineering, School of Computing and IT, Manipal University Jaipur, Jaipur, India; ^5^School of Computing, DIT University, Dehradun, India; ^6^Manipal University Jaipur, Jaipur, India; ^7^Department of Computer Science and Engineering, International Islamic University Chittagong, Chittagong, Bangladesh

## Abstract

Recently, long short-term memory (LSTM) networks are extensively utilized for text classification. Compared to feed-forward neural networks, it has feedback connections, and thus, it has the ability to learn long-term dependencies. However, the LSTM networks suffer from the parameter tuning problem. Generally, initial and control parameters of LSTM are selected on a trial and error basis. Therefore, in this paper, an evolving LSTM (ELSTM) network is proposed. A multiobjective genetic algorithm (MOGA) is used to optimize the architecture and weights of LSTM. The proposed model is tested on a well-known factory reports dataset. Extensive analyses are performed to evaluate the performance of the proposed ELSTM network. From the comparative analysis, it is found that the LSTM network outperforms the competitive models.

## 1. Introduction

With exponential growth in text documents available on Internet, the manual labeling of textual contents in digital form into various classes is extremely challenging to realize. Therefore, many automatic text classification models have been developed such as hierarchical multilabel text classification (HMLTC) [1] and coattention model with label embedding (CMLE) [2]. These models are trained on historical datasets and processed according to a group of labeled data. These models require efficient text encoding models which decompose the text to sequence vectors [1]. The existing text classification models extract a highly discriminative text representation. But these models are generally computationally extensive in nature [2].

Recently, multilabel text classification models were designed. These models are complex compared to single-label classification models [3]. Many researchers have utilized deep learning models for text classification such as recurrent neural network (RNN) and long short-term memory (LSTM). But these models are unable to handle data imbalanced problems [4].

RETRACTED

Recently, many researchers have designed label space dimension reduction to classify text with multiple classes. However, the majority of the models have ignored the sequential details of texts and label correlation with the original label space. Thus, labels were assumed to be meaningless vectors [5]. Also, for the classification of long text, there were a lot of redundant details in textual data. This redundant detail may contain some sort of knowledge too. Thus, the classification of long text requires an efficient model [6].

Mostly, the text details are available in unstructured form. Therefore, the extraction of required details from a huge number of documents becomes a challenging problem [7]. In [8], a bidirectional gated temporal convolutional attention network (BGTCAN) was designed. During the extraction of features, this model has utilized a BGTCAN to obtain the bidirectional temporal features. The attention process was also used to distinguish the significance of various while preserving the maximum text features. In [9], an efficient text classification model was proposed. It has integrated the context-relevant features with a multistage attention model by considering TCN and CNN.

In [10], an efficient hybrid feature selection model was designed. Binary poor and rich optimization (HBPRO) was utilized to compute the significant subset of required features. A Naive Bayes classifier was then used for classification. HBPRO is based on people's wealth such as rich and poor in the world. The rich group tries to widen their group gap by computing from those in the poor group. Every solution in the poor group moves towards the global optimal solution in the search space by learning from the rich group. In [11], an in-memory processor for Bayesian text classification was designed by considering a memristive crossbar model. Memristive switches were utilized to hold the required details for the text classification. In [12], a hybrid model was proposed. It has integrated the gated attention-based BLSTM and the regular expression-based classifier. BLSTM and an attention layer were utilized to weigh tokens according to their perceived significance and focus on critical fractions of a string.

In [13], a backdoor keyword identification model was proposed to overcome the backdoor attacks with LSTM-based models. In [14], label-based attention for hierarchical multilabel text classification neural network was proposed. An efficient label-based attention module was proposed to obtain significant details from the text using labels from various hierarchy levels. In [15], support vector machines (SVM) were utilized to recognize text and documents.

RETRACTED

From the existing literature, it is found that the LSTM network suffers from the parameter tuning problem. Generally, initial and control parameters of LSTM are selected on a trial and error basis. It means the parameters of LSTM models are selected by manually selecting some possible values. Whichever combination shows better performance is followed as control parameters of LSTM. Parameter tuning deals with the optimization of the control parameters of the LSTM model. It can improve the performance of LSTM, but it comes up with additional computations during the model building time. Therefore, in this paper, an evolving LSTM (ELSTM) network is proposed. The key contributions of this paper are as follows:

1. An evolving long short-term memory (LSTM) (ELSTM) network is proposed for text classification.
2. Multiobjective genetic algorithm (MOGA) is used to optimize the architecture and weights of LSTM.
3. The proposed model is tested on a well-known factory reports dataset. Extensive analyses are performed to evaluate the performance of the proposed ELSTM network.

The remaining paper is organized as follows.  Section 2 discusses the related work.  Section 3 presents the proposed ELSTM network for text classification.  Section 4 presents the performance analysis of the proposed ELSTM network on a well-known factory reports dataset.  Section 5 concludes the paper.

## 2. Related Work

In [16], a bidirectional LSTM (BiLSTM) was proposed for text classification. The word embedding vectors and BiLSTM were utilized to obtain both the succeeding and preceding context information. Softmax was also utilized to obtain classification results. In [17], an attention LSTM (ALSTM) network was proposed for text data classification. The ALSTM has shown significant performance in terms of generalization. In [18], deep contextualized attentional bidirectional LSTM (DCABLSTM) was proposed. By utilizing the contextual attention mechanism, DCABLSTM has the ability of learning to attend to the valuable knowledge in a string. In [19], two hidden layers-based LSTM model (THLSTM) was proposed. The first layer was utilized to learn the strings to demonstrate the semantics of tokens with LSTM. The second layer has encoded the relations of tokens. In [20], a recurrent attention LSTM (RALSTM) was proposed to iteratively evaluate an attention region considering the key sentiment words. Attention and number of tokens were minimized in an efficient manner. The TSLSTM leveraged the coefficients of tokens for classification. A joint loss operator was also used to highlight significant attention regions and keywords. In [21], CNN and LSTM were combined for better performance. It has been found that the integrated model can outperform many competitive models. In [22], LSTM fully convolutional network (LSTMFCN) and attention LSTM-FCN (ALSTMFCN) were designed. The fully convolutional block with a squeeze-and-excitation block was used to improve the performance. These models require significantly lesser preprocessing. In [23], convolutional LSTM (CLSTM) network was designed. CLSTM has been found to be adaptable in evaluating big data, keeping scalability. Additionally, CLSTM was free from any specific domain. However, [16–23] are sensitive to its initial parameters.

RETRACTED

To overcome parameter sensitivity issues with LSTM variants, in [24], particle swarm optimization (PSO) was utilized to optimize the LSTM model. PSO was utilized to tune the initial and control parameters of the LSTM network. It has been found that the PSO-based LSTM achieves remarkable results. In [25], a genetic algorithm was utilized to optimize the LSTM. This model can automatically learn the features from sequential data. In [26], a genetic algorithm was utilized to compute the epoch size, number of layers, units size in every layer, and time window size. However, [24–27] suffer from the stuck in local optima and poor convergence speed issues.

It is found that the LSTM network suffers from the parameter tuning problem. The initial and control parameters of LSTM are generally selected on a trial and error basis. Therefore, in this paper, an ELSTM network is proposed.

## 3. Proposed Methodology

This section discusses the proposed ELSTM model. Initially, LSTM is discussed. Thereafter, MOGA is presented. Finally, MOGA-based LSTM, i.e., ELSTM is discussed.  Figure 1 shows the diagrammatic flow of the proposed model. Initially, the dataset is loaded, and preprocessing operation is applied to it.

Since the data is textual in nature, therefore, word encoding is used to convert the strings to numeric sequences. Finally, the proposed ELSTM is trained on the dataset by using a word embedding layer.

### 3.1. LSTM Network

LSTM is a special kind of variant of recurrent neural network (RNN). It was proposed to overcome the long dependency period problem with RNN. Thus, it can preserve information for a longer period.

Consider a sequence input *S*=*s*_1_, *s*_2_, *s*_3_,…, *s*_*p*_, *s*_1_, *s*_2_, *s*_3_,…, *s*_*p*_ showing each token in the textual data. Mathematically, LSTM can be computed as follows:

(1) $$\begin{array}{c} f_{k}=\sigma \left(W_{f}\cdot i_{k-1}+W_{f}\cdot s_{k}+b_{f}\right), \end{array}$$

where *σ* shows a sigmoid function. *W* and *s* represent the weight matrices and bias vector attributes. *i*_*k*_ is the hidden state and can be computed as

(2) $$\begin{array}{c} i_{k}=\sigma \left(W_{i}\cdot i_{k-1}+W_{i}\cdot s_{k}+b_{i}\right). \end{array}$$

The current layer's memory $\left(\tilde{M}\right)$ can be computed as

(3) $$\begin{array}{c} \tilde{M}=\text{tanh}\left(W_{c}\cdot i_{k-1}+W_{c}\cdot s_{k}+b_{c}\right). \end{array}$$

For *k*^*th*^ token, the memory cell (*C*_*k*_) block can be computed as

(4) $$\begin{array}{c} C_{k}=f_{k}\cdot C_{k-1}+i_{k}\cdot \tilde{M}. \end{array}$$

The activation vector (*o*_*k*_) of the output gate can be computed as

(5) $$\begin{array}{c} o_{k}=\sigma \left(W_{o}\cdot i_{k-1}+W_{o}\cdot s_{k}+b_{o}\right). \end{array}$$

The output vector so-called hidden state vector (*i*_*k*_) can be computed as

(6) $$\begin{array}{c} i_{k}=o_{k}\cdot \text{tanh}\left(C_{k}\right). \end{array}$$

RETRACTED

### 3.2. Fitness Function

The main objective of this paper is to optimize the architecture in such a way that it achieves better performance with less number of hidden layers for the LSTM network [28–30]. Therefore, a multiobjective fitness function is designed by using validation accuracy (*A*_*c*_) and the number of hidden nodes of LSTM. The fitness function (*f*(*t*)) can be defined as

(7) $$\begin{array}{c} f\left(t\right)=\left\{\begin{array}{c} \text{Maximize}\left(V_{A}\right),\\ \text{Minimize}\left(H_{N}\right). \end{array}\right. \end{array}$$

Here, *V*_*A*_ shows the validation accuracy. *H*_*N*_ shows the number of hidden nodes used by the LSTM network.

### 3.3. Multiobjective Genetic Algorithm

This section discusses the MOGA-based LSTM (ELSTM) network. Since (7) is a Pareto optimal problem, Algorithm 1 shows step-by-step procedure of the optimization of LSTM.

The genetic algorithm contains a group of operators to optimize the given fitness function [31, 32]. Initially, the normal distribution is used to obtain the random population. These random solutions act as initial parameters of the LSTM network [33–35]. Fitness function (see Eq. mop) is then used to evaluate the fitness of the computed solutions. Nondominated sorting is then used to rank the solutions. Mutation and crossover operators are then utilized to compute the child solutions [36–39]. Mutation and crossover operators are used to obtain child solutions from the parent solutions for evolving process of genetic algorithms. The nondominated solution with a better trade-off between validation accuracy and the number of hidden nodes is used as a final solution for LSTM.  Algorithm 2 shows the step-by-step procedure of the MOGA-based LSTM network.

RETRACTED

## 4. Performance Analysis

The experiments are performed using MATLAB 2021a software on GPU. Experiments are performed on benchmark factory reports dataset.

### 4.1. Dataset

In this paper, the experiments are performed on a well-known factory reports dataset. It consists of around 500 reports with various textual features such as textual information of the attributes and categorical label.  Figure 2 shows the snapshot of the first eight rows of the dataset. Thus, the dataset contains description, category, urgency, resolution, and cost.

Figure 3 shows the histogram distribution of the target classes. There is a total of four target classes, i.e., electronic failure, leak, mechanical failure, and software failure. It is found that the mechanical failure has a higher frequency than the others. Also, the software failures are significantly lesser than the other failures.

Figure 4 shows the histogram distribution of the string tokens. It is found that the majority of the documents have lesser than ten string tokens. Therefore, we have truncated the strings to have length ten.

Figures 5 and 6 demonstrate the frequently utilized words in the training and validation dataset fractions, respectively. Wordcloud in MATLAB is used for visualization purposes. It shows the various words which are frequently, moderately, and least utilized in the factory reports dataset.

Figures 7 shows the training analysis of the LSTM network when the Adam optimizer is utilized. It has received 89.58% validation accuracy. The epoch and iteration-wise mini-batch training and validation accuracy analysis along with respective losses and base learning rate are shown in Figure 8. From both Figures 7 and 8, it is found that the Adam optimizer-based LSTM suffers from the overfitting issue.

Figures 9 shows the training analysis of the LSTM network when the RMSprop optimizer is utilized. It has received 91.67% validation accuracy. The epoch and iteration-wise mini-batch training and validation accuracy analysis along with respective losses and base learning rate are shown in Figure 10. From both Figures 9 and 10, it is found that the RMSprop optimizer-based LSTM achieves better validation accuracy and validation loss than the Adam optimizer-based LSTM. But RMSprop optimizer-based LSTM still suffers from the overfitting issue.

Figures 11 shows the training analysis of the proposed ELSTM network when RMSprop optimizer is utilized. It has received 95.83% validation accuracy. The epoch and iteration-wise mini-batch training and validation accuracy analysis along with respective losses and base learning rate are shown in Figure 11. From both Figures 11 and 12, it is found that the proposed ELSTM achieves better validation accuracy and validation loss than the Adam optimizer and RMSprop-based LSTM networks. The proposed ELSTM is least affected by the overfitting issue.

RETRACTED

## 5. Conclusion

From the extensive review, it has been found that the LSTM network suffers from the parameter tuning problem. Initial and control parameters of LSTM have been selected purely on a trial and error basis. To overcome this issue, an ELSTM network has been proposed. MOGA was utilized to optimize the architecture and weights of LSTM. The proposed model has been tested on a well-known factory reports dataset. Extensive analyses have been performed to evaluate the performance of the proposed ELSTM network. From the comparative analysis, it has been found that the LSTM network outperforms the competitive models. Compared to the LSTM variants, the proposed ELSTM network achieves approximately 4.2389% validation accuracy.

## Figures and Tables

**Figure 1:** Histogram distribution of the target classes.

**Figure 2:** Screenshot of the factory reports dataset.

**Figure 3:** Histogram distribution of the target classes.

**Figure 4:** Histogram distribution of the string tokens.

**Figure 5:** Frequently utilized words in the training dataset.

**Figure 6:** Frequently utilized words in the validation dataset.

**Figure 7:** Training and validation analysis of the Adam optimizer-based LSTM network.

**Figure 8:** Epoch and iteration-wise mini-batch training and validation accuracy analysis of the Adam optimizer-based LSTM network along with respective losses and base learning rate.

**Figure 9:** Training and validation analysis of the RMSprop optimizer-based LSTM network.

**Figure 10:** Epoch and iteration-wise mini-batch training and validation accuracy analysis of the RMSprop optimizer-based LSTM network along with respective losses and base learning rate.

**Figure 11:** Training and validation analysis of the proposed ELSTM network.

**Figure 12:** Epoch and iteration-wise mini-batch training and validation accuracy analysis of the proposed ELSTM network along with respective losses and base learning rate.

**Algorithm 1:** Optimization of LSTM.

**Algorithm 2:** Evolving long short-term memory networks.

## Data Availability

The data collected during the data collection phase are available from the corresponding author upon request.

## References

[1] Ma Y., Liu X., Zhao L., Liang Y., Zhang P., Jin B. (2022). Hybrid embedding-based text representation for hierarchical multi-label text classification. *Expert Systems with Applications*.

RETRACTED

[2] Liu M., Liu L., Cao J., Du Q. (2021). Co-attention network with label embedding for text classification. *Neurocomputing*.

[3] Xiao Y., Li Y., Yuan J., Guo S., Xiao Y., Li Z. (2021). History-based attention in seq2seq model for multi-label text classification. *Knowledge-Based Systems*.

[4] Jang J., Kim Y., Choi K., Suh S. (2021). Sequential targeting: a continual learning approach for data imbalance in text classification. *Expert Systems with Applications*.

[5] Liu H., Chen G., Li P., Zhao P., Wu X. (2021). Multi-label text classification via joint learning from label embedding and label correlation. *Neurocomputing*.

[6] Deng J., Cheng L., Wang Z. (2021). Attention-based bilstm fused cnn with gating mechanism model for Chinese long text classification. *Computer Speech & Language*.

[7] Tian D., Li M., Shi J., Shen Y., Han S. (2021). On-site text classification and knowledge mining for large-scale projects construction by integrated intelligent approach. *Advanced Engineering Informatics*.

[8] Ren J., Wu W., Liu G., Chen Z., Wang R. (2021). Bidirectional gated temporal convolution with attention for text classification. *Neurocomputing*.

[9] Liu Y., Li P., Hu X. (2022). Combining context-relevant features with multi-stage attention network for short text classification. *Computer Speech & Language*.

[10] Thirumoorthy K., Muneeswaran K. (2021). Feature selection using hybrid poor and rich optimization algorithm for text classification. *Pattern Recognition Letters*.

[11] Viswakumar A., Ganganaik P. B., Raj P. M. P., Rao B. P., Kundu S. (2021). Memristor-based in-memory processor for high precision semantic text classification. *Computers & Electrical Engineering*.

[12] Li X., Cui M., Li J., Bai R., Lu Z., Aickelin U. (2021). A hybrid medical text classification framework: integrating attentive rule construction and neural network. *Neurocomputing*.

[13] Chen C., Dai J. (2021). Mitigating backdoor attacks in lstm-based text classification systems by backdoor keyword identification. *Neurocomputing*.

[14] Zhang X., Xu J., Soh C., Chen L. (2022). La-hcn: label-based attention for hierarchical multi-label text classification neural network. *Expert Systems with Applications*.

[15] Luo X. (2021). Efficient English text classification using selected machine learning techniques. *Alexandria Engineering Journal*.

[16] Liu G., Guo J. (2019). Bidirectional lstm with attention mechanism and convolutional layer for text classification. *Neurocomputing*.

[17] Ouyang Z. S, Yang X. T, Lai Y. (2021). Systemic financial risk early warning of financial market in China using attention-lstm model. *The North American Journal of Economics and Finance*.

RETRACTED

[18] Jiang L., Sun X., Mercaldo F., Santone A. (2020). Decab-lstm: deep contextualized attentional bidirectional lstm for cancer hallmark classification. *Knowledge-Based Systems*.

[19] Rao G., Huang W., Feng Z., Cong Q. (2018). Lstm with sentence representations for document-level sentiment classification. *Neurocomputing*.

[20] Zhang Y., Wang J., Zhang X. (2021). Conciseness is better: recurrent attention lstm model for document-level sentiment analysis. *Neurocomputing*.

[21] Er M. B., Isik E., Isik I. (2021). Parkinson’s detection based on combined CNN and LSTM using enhanced speech signals with v. *Biomedical Signal Processing and Control*.

[22] Karim F., Majumdar S., Darabi H., Harford S. (2019). Multivariate lstm-fcns for time series classification. *Neural Networks*.

[23] Behera R. K., Jena M., Rath S. K., Misra S. (2021). Co-lstm: convolutional lstm model for sentiment analysis in social big data. *Information Processing & Management*.

[24] Kim T. Y., Cho S. B. (2021). Optimizing cnn-lstm neural networks with pso for anomalous query access control. *Neurocomputing*.

[25] Shahid F., Zameer A., Muneeb M. (2021). A novel genetic lstm model for wind power forecast. *Energy*.

[26] Kara A. (2021). Multi-step influenza outbreak forecasting using deep lstm network and genetic algorithm. *Expert Systems with Applications*.

[27] Kumar Shukla P., Kumar Shukla P., Sharma P. (2020). Efficient prediction of drug-drug interaction using deep learning models. *IET Systems Biology*.

[28] Ghosh S., Shivakumara P., Roy P., Pal U., Lu T. (2020). Graphology based handwritten character analysis for human behaviour identification. *CAAI Transactions on Intelligence Technology*.

[29] Hu G., Chen S.-H. K., Mazur N. (2021). Deep neural network-based speaker-aware information logging for augmentative and alternative communication. *Journal of Artificial Intelligence and Technology*.

[30] Kaur M., Singh D. (2021). Multiobjective evolutionary optimization techniques based hyperchaotic map and their applications in image encryption. *Multidimensional Systems and Signal Processing*.

[31] Roostapour V., Neumann A., Neumann F. (2020). Evolutionary multi-objective optimization for the dynamic knapsack problem. https://arxiv.org/pdf/2004.12574.pdf.

[32] Kaur M., Singh S., Kaur M. (2021). Computational image encryption techniques: a comprehensive review. *Mathematical Problems in Engineering*.

[33] Basavegowda H. S., Dagnew G. (2020). Deep learning approach for microarray cancer data classification. *CAAI Transactions on Intelligence Technology*.

[34] Xu Y., Qiu T. T. (2021). Human activity recognition and embedded application based on convolutional neural network. *Journal of Artificial Intelligence and Technology*.

RETRACTED

[35] Singh D., Kumar V. (2019). Image dehazing using moore neighborhood-based gradient profile prior. *Signal Processing: Image Communication*.

[36] Xue X., Lu J., Chen J. (2019). Using NSGA‐III for optimising biomedical ontology alignment. *CAAI Transactions on Intelligence Technology*.

[37] Gupta B., Tiwari M., Singh Lamba S. (2019). Visibility improvement and mass segmentation of mammogram images using quantile separated histogram equalisation with local contrast enhancement. *CAAI Transactions on Intelligence Technology*.

[38] Jiang D., Hu G., Qi G., Mazur N. (2021). A fully convolutional neural network-based regression approach for effective chemical composition analysis using near-infrared spectroscopy in cloud. *Journal of Artificial Intelligence and Technology*.

[39] Singh D., Kumar V. (2018). A novel dehazing model for remote sensing images. *Computers & Electrical Engineering*.

